This article has been retracted.

# Biodegradation modeling of phenol using *Curtobacterium flaccumfaciens* as plant-growth-promoting bacteria

**DOI:** 10.1016/j.heliyon.2022.e10490

**Published:** 2022-09-02

**Authors:** Khaled Khleifat, Mousa Magharbeh, Moath Alqaraleh, Mutaz Al-Sarayrah, Ibrahim Alfarrayeh, Yaseen Al Qaisi, Ahmad Alsarayreh, Mohammad Alkafaween

**Affiliations:** a Faculty of Allied Medical Sciences, Al-Ahliyya Amman University, Amman, Jordan; b Department of Pharmaceutical Chemistry, Faculty of Pharmacy, Mutah University, Al-Karak 61710, Jordan; c Pharmacological and Diagnostic Research Center, Faculty of Pharmacy, Al-Ahliyya Amman University, Amman, Jordan; d Department of Biological Sciences, Faculty of Science, Mutah University, 61710 Al-Karak, Jordan; e Department of Applied Biology, Faculty of Science, Tafila Technical University, 66110 Tafila, Jordan; f Faculty of Pharmacy, Department of Pharmacy, Al-Zaytoonah University of Jordan, Amman, Jordan

**Keywords:** Phenol, Biodegradation, Biodegradation pathway, *Curtobacterium flaccumfaciens*

## Abstract

Phenol is a major worry pollutant resulting from industrialized manufacturing and chemical reactions. The growth kinetics and biodegradation of phenol were initially investigated using *C. flaccumfaciens*, a recently identified plant growth stimulating bacterium. Based on the Haldane inhibition model, Haldane's growth kinetics inhibition coefficient (Ki), half-saturation coefficient (Ks), and the maximum specific growth rate (max) for phenol-dependent growth kinetics were estimated to be 329 (mg/L), 9.14 (mg/L), and 1.05 (h^−1^), respectively. With a sum of squared error (SSR) of 1.36 × 10^−3^, the Haldane equation is well adapted to empirical data. The improved Gombertz model also accurately predicts phenol biodegradation trends. The rate of phenol biodegradation and the lag time both increased as the initial phenol concentrations were increased. *C. flaccumfaciens* growth and phenol biodegradation were best achieved at a pH of 7.0 at a temperature of 28 °C incubation. A phenol biodegradation mechanism by *C. flaccumfaciens* has been proposed. In conclusion, this study revealed the ability of *C. flaccumfaciens* to promote plant growth and biodegrade phenol simultaneously. This could aid in rhizoremediation and crop yield preservation in phenol-stressed conditions.

## 1 Introduction

Organic hydrocarbons are mostly pollutants that contain a diverse range of substances that can be dangerous to human health. Phenol and its derivatives are commonly utilized as beginning materials in industrial and agricultural production and are termed secondary byproducts [1]. Phenol is harmful to a variety of aquatic organisms at lower doses of mg/L, and it leads to olfactory and taste issues in water [2, 3, 4]. Excess phenol exposure causes problems with the central nervous system, paralysis, liver failure, loss of appetite, rashes, difficulty speaking, digestive problems, vomiting, morbidity, weight loss, and cancer [3, 5]. It has a deadly effect due to its fast penetration and cutaneous imbibition, inhalation, and consumption [6, 7, 8]. It has the potential to cause severe respiratory and ocular discomfort. It's classified as a human carcinogen, and at low quantities (5–25 mg/L), it can kill fish. Because of the widespread usage of phenol in the United States, as well as its inherent toxicity, the US Environmental Protection Agency designated phenol as a primary concern pollutant [9].

The environmental disposal of phenol is facing further exacerbations as a result of economic burdens or more harmful by-products [10, 11, 12, 13]. Solvent extraction, absorption, ion exchange, incineration, chemical activated carbon absorption, oxidation, oxidation, and liquid extraction have all been reported as successful methods for removing phenol chemicals. However, both chemical and physical procedures are frequently costly, and most of these treatments fail to fulfill the goal of phenol breakdown, instead of converting it to a different phase, resulting in pollution and hence harmful by-products. Biodegradation of phenol, on the other hand, is a more cost-effective and environmentally beneficial option. As a result, the relevance of biological phenol treatment has become an escalation process for pollution control [14, 15, 16].

Plant growth-friendly bacteria have been used to resurrect agricultural crop output for decades [17, 18, 19]. Plants benefit from these microorganisms in a variety of ways, including increasing nutrient bioavailability and biosorption, reducing soil-plant pathogens by controlling pathogenic factors, constructing materials that support plant growth, and removing injurious constituent parts from the soil, such as detrimental compounds that may interrupt the growth of plants [20, 21]. PGPB (Plant growth-promoting bacteria) are a type of microbe that can be used instead of chemical fertilizers, insecticides, as well as plants that have been genetically engineered. Furthermore, PGPB can counteract the negative impacts of environmental stressors in soils. High salt concentrations [22, 23], pollution by heavy metals as well as other non-living pollutants, or different organic contaminants [17, 24, 25] are all sources of stress. As a result, PGPB purposes as a likely mean in the re-establishment of agricultural fields which were previously unsuitable for fodder or sustenance. Many organic molecules, such as phenol, are resistant to mineralization, resulting in environmental issues. As a result, it turns out to be essential to take care of manufacturing wastes for the proper phenol removal from the surroundings to preserve the soil and aquatic ecosystems' capability and integrity [11, 26, 27, 28, 29, 30].

For many decades, scientists have been fascinated by the biodegradation of aromatic chemicals such as phenol [31, 32, 33]. Bacterial cells are always evolved to use unprocessed organic compounds produced by people and are found in a variety of habitats [7, 34, 35]. Because of its complete biodegradation and low cost, bioremediation or biodegradation is the best option in general. The goal of this study was to see if isolated growth-promoting *C. flaccumfaciens* could biodegrade phenol, which was validated by GC-MS and HPLC analyses. This involved modeling of *C. flaccumfaciens* growth kinetics utilizing phenol as a carbon and energy source.

## 2 Materials and methods

### 2.1 Bacterial strain

*C. flaccumfaciens* was the bacterial strain used in this study. *C. flaccumfaciens* was isolated from Jordan. It was identified by Anna Rosa Sprocati of Rome, Italy, using 16S rRNA methods. The accession number for its nucleotide sequence in Genbank was (MN083287). The biochemical identification was double-checked using the REMEL RapID™ ONE System (Thermo Scientific™, Catalog number: R8311006) and REMEL RapID NF Plus systems (Thermo Scientific™, Catalog number: R8311005). it was also examined using a microscope for the morphological characteristics.

### 2.2 Media and culture conditions

#### 2.2.1 Preparation of mineral media with phenol

Three solutions were produced individually to prepare this media: (a) A phenol solution was made by dissolving 5 g of phenol (Sigma-Aldrich) in 200 mL of deionized water (the final concentration was 25,000 ppm). This solution was filter-sterilized to exclude any potential thermal effects on the phenol. (b) Mineral media have been prepared by combining the materials in a 1000 mL Erlenmeyer flask: one gram of K_2_HPO_4_ and NH_4_NO_3_, 0.5 g of (NH_4_)_2_SO_4_, MgSO_4_, KH_2_PO_4,_ and NaCl, 0.02 g of CaCl_2_ and FeSO_4_ (Sigma-Aldrich). After that, the media was autoclaved in flasks holding the requisite amount of mineral broth medium and the required concentration of phenol. Wolfe’s mineral solution was made by dissolving 1.5 g of nitrilotriacetic acid (Thermo Scientific™) in 500 mL of deionized water, the pH was set to 6.5 by adding KOH to achieve the highest solubility. Then the subsequent were added: 3 g of MgSO_4_.7H_2_O, 1g of NaCl, 0.5 g of MnSO_4_. H_2_O, 1 g of FeSO_4_.7H_2_O, 0.1 g of CoCl_2_.6H_2_O, CaCl_2_ and ZnSO_4_.7H_2_O, 10 mg of CuSO_4_.5H_2_O (Sigma-Aldrich). The masses of AlK(SO_4_)_2_.12H_2_O, H_3_BO_3_, and Na_2_MoO_4_.2H_2_O (Sigma-Aldrich) are all 10 mg. The bottle was therefore filled to the mark with distilled water and forcefully shaken before being sterilized with a filter. Lastly, the phenol-containing mineral broth media was completed by filling each flask with 0.5 mL Wolfe's with the appropriate amount of phenol according to the phenol concentration needed. For example, 0.5 and 0.4 mL of Wolfe's and phenol solutions, respectively were added to 49.1 mL of mineral media to attain a phenol concentration of 200 ppm.

#### 2.2.2 Assessment of growth on phenol

*C. flaccumfaciens'* ability to grow on phenol as a sole carbon source was evaluated by culturing it in TSB towards the mid of log phase (OD_600_ = 0.50). The cells of bacteria were collected by centrifugation for 15 min at 4000 rpm. At 600 nm, the OD was set to 0.20, and the cells were washed and suspended in a mineral medium to be employed as an inoculum later. *C. flaccumfaciens* was inoculated into mineral media with a phenol content of 700 ppm. Spectrophotometry at 600 nm was used to track bacterial growth for 12, 24, 36, 48, 60, 72, 84, and 96 h. For the control, the same approach was used (mineral media containing 700 ppm phenol, uninoculated).

#### 2.2.3 Plant growth-promoting characteristics

Salkowski's reagent creates a pink complex when it comes into touch with Indole-3-acetic acid (IAA); a positive reaction shows that bacteria may convert L-tryptophan to IAA or linked chemicals [36]. A carboxylic acid IAA is a plant growth hormone in the auxin family that stimulates branching and root formation. Phosphate solubility was evaluated using an inorganic phosphorous medium of Pikovskaya (PKO) at 30 °C and checked each day for seven days. The potential to solubilize phosphate is indicated by the presence of a clear halo around colonies. The creation of siderophores was investigated using agar plates of chrome azurol S (CAS), and the existence of siderophores is indicated by a shift in color of the colony's surroundings from blue to orange [37]. A nitrogen-free medium was used to assess *C. flaccumfaciens’* ability for nitrogen fixation. After washing twice, cultures of *C. flaccumfaciens* grown overnight in Trypticase Soy Broth (TSB) media were re-suspended in saline phosphate buffer (PBS), pH 7.4. The bacterium concentration was adjusted to an OD_600_ of 0.50. A 30 μL aliquot of bacterial suspension was injected into 10-milliliter tubes containing 4 ml of New Fabian broth (NFb) and incubated at 28 °C. After 72 h of incubation on the culture media, a sub-surface pellicle was formed to ensure the growth of bacteria [38]. The ability of nitrogen fixation was demonstrated by repeated re-growing in NFb media. The procedures have been carried out in triplicate in every case.

#### 2.2.4 Estimation of phenol

Phenol concentration was determined using the 4-aminoantipyrine spectrophotometric method [39]. 0.5 N of ammonium hydroxide (Thermo Scientific™) was added and thoroughly mixed. The pH of 7.9 was adjusted by applying potassium phosphate (KH_2_PO_4_) buffer, and pH (6.8) was achieved by adding 2 and 8 percent as w/v of 4-aminoantipyrine (Sigma-Aldrich) and potassium ferricyanide (Fluka), respectively. To complete the reaction, the specimens were left at room temperature for 15 min before measuring the absorbance at 510 nm with a UV–Vis Spectrophotometer. A standard calibration curve was created using a spectrophotometer to determine the amount of phenol based on the obtained absorbance.

#### 2.2.5 Correlation between growth conditions and degradation of phenol

The potential of *C. flaccumfaciens* to break down a 700 ppm phenol was investigated in a mineral medium. *C. flaccumfaciens* was cultivated in the mineral media under various conditions using a shaking incubator. The potential effect of pH on phenol degradation by *C. flaccumfaciens* cells was scrutinized using different values of pH (5.5, 7, 8, and 9). The impacts of 25, 28, 33, and 37 °C on *C. flaccumfaciens* phenol degrading potential were also investigated. The percentage of removal was approximated at the moment using a fixed length (48 h) to remove any mistakes that resulted from the varying extents of the setback stages, the challenges in determining the time needed to attain full degradation, or if the degradation had stalled. This is because many cells exhibited no further phenol degradation as time progressed, or it represents the elapsed time between each evaluation [11].

#### 2.2.6 HPLC analysis

In this experiment, a Shimadzu LC-10A HPLC/UV-Vis detector (Shimadzu, LC-10A, Tokyo, Japan) and a Luna C18 column (4.6 × 250 mm, 5 m, 100) were utilized. The measurement of phenol compound concentration was performed at 30 °C in a column compartment with temperature control. “The mobile phase was composed of 0.1 percent acetic acid (solvent A) and 1:1 v/v % (acetonitrile/methanol) (solvent B), with the following parameters: 0.1–1 min, 95 % confidence A; 1–6 min, 50 percent A; 6–10 min, 5 percent A. The UV detector had a capacity of 10 L and a flow rate of 1.0 mL/min (280 nm). To validate the biodegradation of phenol, samples of culture media containing 700 ppm phenol were analyzed at various time intervals (0, 12, 24, 48, 72, and 96 h)” [40].

#### 2.2.7 GC-MS analysis

After 96 h of incubation for the cultured phenol-containing medium and the control, 30 ml was taken from each flask and stabilized with 4.5 ml of a 10% CuSO_4_ solution. After that, the pH was adjusted with 2 drops of concentrated H_3_PO_4_. Both stabilized samples were then extracted with 2 ml of dichloromethane, dried with anhydrous Na_2_SO_4_, and pre-concentrated using rotary evaporation. For GC-MS analysis, the resulting residue was dissolved in 5 ml methanol. The GC-MS analysis was performed using a Varian Chrompack CP-3800 GC-MS-200 (Saturn) equipped with a DP-5 (5% diphenyl, 95% dimethyl polysiloxane) GC capillary column (30 m × 0.25 mm i.d., 0.25 m film thicknesses) with helium as the carrier gas at a flow rate of 1 ml/min. The MS temperature source was set to 180 °C and the ionization voltage was set to 70 eV. The column temperature was maintained at 60 °C (isothermal) for 1 min before being elevated to 270 °C at a rate of 3 °C/min. A combination of n-alkane hydrocarbons (C8–C20) was individually examined using the same chromatographic settings and DP-5 column. The GC-MS spectra were manually analyzed according to Das et al [41] and Kumar et al [42]. “The injector temperature was set to 270 °C and the interface temperature was Kept at 280 °C. Electron ionization (EI) mass spectra with a range of 35–650 (m/z) were recorded in fully scanned mode at an electron energy of 70 eV. The phenolic degradation metabolites were identified by comparing their retention time (RT) in minutes and mass spectra with the National Institute of Standards and Technology (NIST) library, USA/Wiley, or by comparing the RT with accessible authentic standards” [40].

#### 2.2.8 Method for the assurance and validation of analytical quality

To verify linearity, “four injections of phenol at five different concentrations (50, 250, 500, 1000, and 1500 ppm) were used. The R^2^ value of 0.996 for phenol demonstrated excellent linearity. In order to calculate the limit of detection (LOD) and limit of quantitation (LOQ), the standard solution was diluted until the signal-to-noise ratio (S/N) corresponded to three and ten, respectively. The LOD and LOQ values were 2.45 and 8.17 ppm, respectively. A relative standard deviation (RSD) of 2.7 indicates that a very precise result was obtained. For the improvement test, blank samples were spiked with known concentrations of phenol standard solution (50, 500, and 1500 ppm). For the phenol component, all recovery results at various concentrations ranged from 83 to 106 percent” [40].

#### 2.2.9 Mathematical methods

Typically, the logistic equation (Equation 1) is employed to characterize the growth profile of biomass in a batch reactor for both exponential and stationary phases. The logistic equation is expressed using the differential formula:

(1) $$\frac{dX}{dt}=\mu_{m}X\left(1-\frac{X}{X_{m}}\right)$$

where *μ*_*m*_ is the greatest rate of specific growth (hr^−1^) achievable in a particular atmosphere and *X*_*m*_ is the highest cell density attainable in those surroundings (OD_600_). The following formula for cell density (Equation 2) is obtained by integrating the logistic equation:

(2) $$X=\frac{X_{o}e^{\mu_{m}t}}{1-\left(\frac{X_{o}}{X_{m}}\right)\left(1-e^{\mu_{m}t}\right)}$$

where *X*_*o*_ denotes the primary cells concentration (OD_600_) and *t* is the time. To characterize the relationship between both the specific growth rate *μ* and the amount of substrate *S*, several kinetics models have been devised. The Haldane equation (Equation 3) represents the most commonly used inhibitory expression at greater substrate concentrations and when inhibitor concentration influences growth:

(3) $$\mu =\frac{\mu_{\max}S}{K_{s}+S+\frac{S^{2}}{K_{1}}}$$

Where *μ*_*max*_ is Haldane's maximal specific growth rate (hr^−1^), *K*_*s*_ is the half-saturation coefficient (ppm), and *K*_*I*_ is Haldane's growth kinetics inhibition coefficient (ppm).

All experiments in this study were done in triplicates, and the results were expressed as mean ± standard deviation (SD).

## 3 Results and discussions

### 3.1 PGPB characterization

Only phosphate solubilization and nitrogen fixation have been detected in *C. flaccumfaciens* out of four plant growth supporting traits (Table 1). The nitrogen-fixing process is controlled by the nitrogenase enzyme complex, which is produced by the nif gene. As previously stated, the test involves adding a 2 mL alcoholic solution of 0.5 percent bromothymol blue to NFCC-medium to emphasize the growth of bacterial colonies [43, 44]. Because many necessary elements, including phosphorus, are found in the soil in an unreachable shape, improving phosphorus mobility in the soil and making it accessible for plant growth by freeing it from insoluble or fixed forms is crucial. According to Nautiyal's methods, the potential of the bacterial isolates to mobilize phosphorus was checked using a plate test with agarized and modified Pikovskaya medium (PVK) and bromophenol blue (BPB), which emphasizes and causes the development of even more obvious halos [45, 46]. Individual strains' phosphorus mobilization capacity and efficiency are assessed by selecting microorganisms that produce halos or clear areas on the incubation plate as a result of the generation and release of organic acids around them.

**Table 1:** Features of *C. flaccumfaciens* that promote plant growth.

The similarity of 16S rDNA sequencing (%)	Accession Number	Features that promote plant growth			
		Nitrogen fixation	Siderophore production	Phosphate solubilization	Auxin production
*C. flaccumfaciens* 99%	MN083298	+	-	+	-

### 3.2 Growth of *C. flaccumfaciens* versus phenol degradation

Using *C. flaccumfaciens*, a plant growth-promoting bacterium (Table 1) is investigated for the degradation process of phenol as a sole substrate for growth and energy in the batch process. As part of the SUPREME project, the strain was isolated from soil by the ENEA-Casaccia laboratory. It was stored in the MIRRI-It ENEA microbiological collection. Based on the condensing phenol with 4-aminoantipyrine, the phenol was calculated by measuring the absorbance at 510 nm, which after oxidation reaction with alkaline potassium ferry cyanide, generated the red hue [39]. The quantity of phenol removed by bacteria can thus be measured using the phenol standard curve (not shown). The results showed that after 103 h of incubation, the culture could degrade phenol at the highest concentration of 700 ppm (Figure 1). The results of growth based on OD_600_, on the other hand, agreed with those of biodegradation results (Figure 2).

**Figure 1:** The amount of phenol (ppm) that remained after growing *C. flaccumfaciens* cells on various concentrations of phenol (ppm) as the only carbon and energy source. The growth conditions were 28 °C incubation temperature, 150 rpm shaking rate, and pH 7.0. Each data point is the average of at least three independent experiments with error bars indicating STDEVs (σn-1).

**Figure 2:** *C. flaccumfaciens* cells grown on M9 minimal medium plus different concentrations of phenol (ppm) as only carbon and energy source at 28 °C, shaking rate of 150 rpm, and pH 7.0. Each data point is the average of at least three independent experiments with error bars indicating STDEVs (σn-1).

### 3.3 Effect of substrate concentration

*C. flaccumfaciens* was capable of utilizing phenol as a substrate for obtaining carbon and energy. To investigate the biodegradability of phenol, two types of negative controls were used in all cases: phenol-containing cell-free media and phenol-containing culture that was destroyed by heat. No evidence of phenol biodegradation activity has been found to support the theory that the biodegradation activity is only due to *C. flaccumfaciens* cells. Initially, six different phenol concentration trials were employed (200, 400, 700, 800, 1000, and 1100 ppm) (Figure 1). Raising the phenol content to 700 ppm after 48 h of incubation resulted in the highest percentage of removal (63%) as shown in Table 2. The rate of time deterioration began to slow as phenol concentration was raised. Because increasing the phenol concentration, especially above the threshold, caused the cells to become more repressed. Above 700 mg/mL concentration, competition led to an inhibitory effect on the rate of the chemical reaction. Therefore, the removal percentage of more than 700 mg/mL will be decreased as shown with the lower concentration used (200 and 400 ppm). Moreover, the use of the fixed time (48 h) was “to estimate the percentage removal at that time to avoid any errors caused by the different lengths of the delay phases” [40]. These findings are consistent with prior research on phenol breakdown by microorganisms [6, 47, 48, 49].

**Table 2:** The impact of phenol concentration on the percentage of phenol elimination in *C. flaccumfaciens*. Data was gathered after a 48-hour incubation period.

Concentration (ppm)	Removal (%) (mean ± SD)
200	52 ± 1.56
400	59 ± 1.77
700	63 ± 1.89
800	36 ± 1.08
1000	29 ± 0.87
1200	28 ± 0.84

### 3.4 Kinetic modeling

Using nonlinear regression, the tentative growth biomass patterns at different primary concentrations of phenol were suited to the logistic equation. To determine the model fitting parameters, the Microsoft Excel 2007 (Solver add-in) was used to minimize the SSR. Figure 3 depicts the logistic model characteristics, as well as empirical results, for various initial phenol concentrations. As can be shown, with an initial phenol concentration of 700 ppm, biomass growth approximated the maximum extent of the stationary population. in addition, with a 700 ppm phenol as the initial substrate concentration, the mass of cells had the specific growth at its highest rate (*μ*_*m*_). Growth mass was described as growing at a slower rate and its stationary population size is small at 1200 ppm initial phenol concentration (Figure 3).

**Figure 3:** The effect of phenol concentration on *C. flaccumfaciens* growth rates (h^−1^). Based on OD_600_ assessments, growth curves were made and the rate of growth for bacterial cells grown on every phenol concentration was estimated at the same time. The growth conditions were 30 °C incubation temperature, 150 rpm shaking rate, and pH 7.0.

Plotting the data of biomass growth throughout the log phase resulted in the estimation of the specific growth rate (*μ*) for the various baseline phenol concentrations. The slope produced by graphing *ln(X/X*_*o*_*)* versus time equals the particular growth rate (*μ*). The link between the specific growth rate and the starting phenol concentration was well represented by the Haldane equation (Figure 3 and Table 3). Haldane's parameters were estimated using a non-linear regression technique based on the minimization of SSR (Table 4). The greatest rate of specific growth, half-saturation coefficient, and inhibition of Haldane's growth kinetics coefficient determined from the Haldane equation are 2.28 h^−1^, 4.3, and 291 ppm, respectively. SSR of 2.41 × 10^−3^ was fitted to the experimental data by the Haldane equation. Figure 3 depicts a typical growth kinetics pattern for an inhibiting substrate. The results illustrate that the value of the specific growth rate was raised with rising the concentration of phenol equal to roughly 200 ppm, then begins to decrease as the primary phenol concentration boosts. To simulate phenol degradation, the adapted Gombertz formula (Equation 4) [50] was used:

(4) $$S=S_{o}\left\{1-\exp\left\{-\exp\left[\frac{R_{m}}{S_{o}}e\left(\lambda -t\right)+1\right]\right\}\right\}$$

where *S* denotes the concentration of phenol, *S*_*o*_ is the initial concentration of phenol, *R*_*m*_ is the maximum growth rate, λ is the lag phase time, and *t* is the time (h).

**Table 3:** The logistic model's regression parameters for describing biomass growth variables.

Phenol Concentration (ppm)	$\mu_{m}$ (hr^−1^)	$X_{m}$ (OD_600_)	SSR
200	0.300	0.293	8.11 × 10^−6^
400	0.195	0.270	4.44 × 10^−5^
700	0.065	0.400	7.09 × 10^−3^
800	0.105	0.322	2.66 × 10^−3^
1000	0.202	0.116	7.47 × 10^−5^
1200	0.050	0.101	3.00 × 10^−5^

**Table 4:** Phenol degradation using the parameters of Haldane.

Microbial Strain	$S_{o}$ (ppm)	$\mu_{\max}$ (hr^−1^)	$K_{s}$ (ppm)	$K_{1}$ (ppm)	Reference
*C. flaccumfaciens*	200–1200	2.280	4.3	291	This study
*Bacillus cereus* MTCC 9817	0–2000	0.4396	129.4	637.8	Bai et al., 2007
*Ewingella americana*	100–1000	0.29	5.16	1033.7	Khleifat (2006)
*Alcaligenes faecalis*	10–1400	0.15	2.22	245.37	Der Yang and Humphrey, (1975)
*Mixed culture*	0–800	0.3085	44.92	525.00	Saravanan et al., (2008)
*Pseudomonas* WUST-C1	0–1600	2.500	48.70	100.6	Liu et al., (2013)
*P. putida* (ATCC 17514)	0–500	0.567	2.39	106.0	Wang et al., (1996)
*Pseudomonas citronellolis*	50–1500	0.246	14.85	890	Panigrahyet al., (2020)
*Acinetobacter calcoaceticus*	60–500	0.542	36.2	145.0	Kumaran and Paruchuri, (1999)
*Pseudomonas putida*	25–800	0.900	6.93	284.3	Wang and Loh, (1999)

The revised Gombertz model fits phenol biodegradation trends fairly well. Table 5 shows the model's fitting parameters. When the starting phenol concentrations were increased (up to 700 ppm), the rate of phenol biodegradation and the lag time both increased.

**Table 5:** Parameters obtained for specific degradation rate (*R*_*m*_).

Phenol Concentration (ppm)	$R_{m}$ (mg/L.hr)	λ (hr)
200	5.4	12.1
400	6.7	14.5
700	9.0	10.2
800	9.4	18.3
1000	9.2	6.3
1200	10.3	13.1

### 3.5 The impact of reaction temperature on *C. flaccumfaciens*' phenol degradability and growth

After a 48-hour incubation period, the effect of diverse incubation temperatures (25, 28, 33, and 37 °C) on phenol degradation by *C. flaccumfaciens* was examined (Table 6). The adoption of a constant time (48 h) was done to keep away from any inaccuracies reasoned by variations in lengths of the delay phases, as well as the difficulties in understanding how long it would take to attain total degradation or whether it had discontinued. This is for the reason that several cells did not reveal any more phenol breakdown as time passed, or it expresses the elapsed moment for each trial [6, 48].

**Table 6:** The effect of growing conditions on the rate of phenol biodegradation by *C. flaccumfaciens*. After a 48-hour incubation period, data was collected.

Condition	Value	Removal (%)	OD_600_
Incubate temperature (^o^C)	25	35.5 ± 1.10	0.33
	28	63.0 ± 1.89	0.47
	33	42.3 ± 1.24	0.38
	37	24.6 ± 0.94	0.37
pH	5.5	13.5 ± 0.61	0.12
	7.0	63.0 ± 1.89	0.47
	8.0	37.0 ± 1.04	0.35
	9.0	0.00 ± 0.00	0.01

When the minimum medium was supplied with phenol (700 ppm), all temperatures indicated an improvement in bacterial growth based on phenol removal percentage measurements. At the incubation temperature of 28 °C, a significant increase in phenol removal was found, and the best growth was seen. The increased growth yield could be attributed to the phenol basic medium's more effective metabolic turnover of phenol as a carbon source. Above 33 °C, the incubation temperature becomes crucial, and therefore any further rise in incubation temperature causes a significant decrease in the rate of phenol degradation. As a consequence, the biodegradation of phenol appears to be possible at incubation temperatures ranging from 25 °C to 37 °C, with 28 °C being the most preferred incubation temperature for *C. flaccumfaciens* cells.

The metabolic fate of organic contaminants including phenol was affected by variations in incubation temperatures, with the mesophilic temperature providing better conditions for their biodegradation, or this could be due solely to the effect of incubation temperature on the activities of the enzyme(s) involved [6, 47, 48, 49]. It's worth mentioning that the initial temperature can also have a big impact on the degradation of organic pollutants like phenol, sometimes even more than the nutrient availability [11, 51].

Furthermore, each of the biological reactions involved in the breakdown pathway has an optimum temperature and pH, therefore metabolism rates will differ under different conditions [52]. As a result, each bacterial species has its own set of ideal growth temperatures. *Corynebacterium*, for example, has been found to break down phenol at temperatures ranging from 30 to 37 degrees Celsius [53]. At a temperature of 33 °C, *Acetobacter* sp displayed its normal biodegradation of phenol [54].

### 3.6 The influence of media pH on phenol biodegradation

After a 48-hour incubation period, the influence of several pHs (5.5, 7, 8, and 9) on phenol degradation by *C. flaccumfaciens* was examined (Table 6). The biological control in the uncultivated culture was used to determine whether or not the decrease in phenol concentration is due to the chemical reaction and to ensure that the *C. flaccumafaciens* bioactivity will result in a decrease in the final phenol concentration on the culture medium. The tested pH had no effect on the concentration of phenol in the uncultivated culture. However, the varying phenol degradation rates of *C. flaccumfaciens* cells were due to the variable pH values. These variables affected the level of phenol dissipation, which is determined by the pH of the bacterial culture.

These findings revealed that a pH of 7.0 is optimal for maximal phenol breakdown by bacteria. Enzymes that cause *C. flaccumfaciens* cells to degrade phenol may have optimum enzymatic activity at pH 7.0. The ideal pH for the biological degradation of phenol varied by bacterium; for example, pH ranged from 8 to 11 for the bacterium *Halomonas campisalis* [55], whereas pH was 6.8 for the degradability of phenol by *Klebsiella oxytoca* [55, 56]. The optimal pH for *Arthrobacter* to degrade 4-CBA is 6.8. [57]. The optimum pH for *Ewingella americana* to biodegrade phenol was 7.5. The enzymes for phenol degradation by *C. flaccumfaciens* are likely to be at their most active at pH 7.5. Research into microbial phenol breakdown has developed considerably, resulting in the isolation, development, acclimation, and selection of some bacteria that can live solely on organic pollutants for carbon and energy. However, insufficient attempts have been taken to mitigate their harmful influence on the environment [58, 59].

Numerous bacterial species have already been employed in phenol biodegradation investigations that utilize phenol and other aromatics as their sole source of carbon and energy [48, 52]. These include *Bacillus* sp, *Acinetobacter* sp, *Pseudomonas* sp, *Ewingella Americana*, *Achromobacter* sp, [60, 61, 62, 63, 64], *Phanerocheate chrysosporium*, *Streptomyces* sp, *Fusarium* sp, *Ralstonia* sp, and *Corious versicolor* [7, 65]. Physiological parameters are important for any microorganism's development and biodegradation behavior [66, 67], however, maximum growth is only possible when certain physiological characteristics are at their best. Thus, numerous physiological characteristics that commonly interfere with a microbe's biodegradation activity include nutrition availability, incubation temperature, and pH.

### 3.7 HPLC analysis

HPLC was used to examine the samples that had been treated with *C. flaccumfaciens*. At a retention time of 7.5 min, the peak revealed the position of the normal 100 ppm phenol area (Figures 4A-D). The phenol at zero time and the sample treated with *C. flaccumfaciens* after 96 h have maxima at 7.5 and 2.5 min, respectively, as shown in the Figure. The disappearance of the phenol signal at 7.5 min provided more evidence for phenol degradation. The spectrum also indicated a peak at 2.5, which corresponds to catechol, the primary intermediate produced by different microbial strains as a result of phenol metabolism [21].

**Figure 4:** Representative chromatograms for 100 ppm phenol (control) (A); 100 ppm catechol (standard) (B); phenol compound sample at zero time (C); and phenol compound after 96 h’ incubation (D).

### 3.8 GC analysis

In general, bacterial culture biodegraded the phenol compound and demonstrated two reaction mechanisms. In the first step, the hydroxylase enzyme converted phenol to catechol by using molecular oxygen. Catechol was hydrolyzed by 1,2-dioxygenase in the second stage to produce cis, cis-muconic acid via the ortho route and/or through the meta-pathway using 2,3-dioxygenase [68]. The GC-MS chromatograms for the inspected sample comprise more than seven peaks with differentiated retention times (Figure 5). The NIST mass spectral database identified the following degradation and condensation products of catechol and/or phenol in the GC-MS analysis of these main peaks (Figure 6): The coupling of phenol and catechol [1,1'-biphenyl]-2,2',3,3'-tetrol (1) at (RT = 11.80min, and m/z = 220.3), as demonstrated in Figure 6. On other hand, the condensation of the acetaldehyde with phenol and/or catechol produced 4-(1-hydroxy-1-phenylethyl) phenol (2) at (RT = 12.436 min, and m/z = 214.4), and (3) at (RT = 22.806 min, and m/z = 431.8) as demonstrated in Figure 6. The following product of the condensation of the propanal with phenol and/or catechol produced 3,3'-(1-hydroxypropane-1,1-diyl) di(benzene-1,2-diol) (4) at (RT = 18.319 min and m/z = 277.3), 2-[1-hydroxy-1-(2-hydroxyphenyl)propyl]-6-(1-hydroxypropyl)phenol (5) at (RT = 21.642 min and m/z = 297.6) and 4,4'-(1-hydroxypropane-1,1-diyl)diphenol (6) at (RT = 27.478 min and m/z = 245.5) and other condensation and elimination products such as, 3-(3,4-dihydroxyphenyl)-2-hydroxypropanoic acid (7) at (RT = 16.730 min and m/z = 197.3) (Figure 6), all those products from degradation and condensation confirm that catechol cleavage through meta pathway (catechol-2,3-dioxygenase).

**Figure 5:** The GC-MS chromatograms (A) control (phenol) (B) standard (catechol) and (C) sample.

**Figure 6:** The potential chemical structures for anticipated molecules, as well as the fragmentation pattern of the important peaks identified in the GC-MS analysis (1–7).

The analysis of the phenol control sample (RT = 5.099 min, and *m/z* = 94.0), and a standard sample of catechol at (RT = 8.194 min and *m/z* = 110.3) are shown in Figure 7. On the other hand, the investigation of GC-MS for the extractable yield sample of bacterial culture (Figure 6) demonstrated that the hydroxylase enzyme converted the most phenol molecule to catechol in the first step, employing molecular oxygen to do so [68, 69]. All of the products of this pathway undergo additional oxidation steps to generate acetaldehyde and pyruvate via the meta pathway, which are subsequently decomposed to CO_2_ and H_2_O. Due to *C. flaccumfaciens'* rapid utilization of these compounds, it was difficult to detect them in this study. According to the phenol degradation pathway, which is shown in Figure 8, catechol, acetaldehyde, and propanal can be produced from the degradation of phenol as a substrate, resulting in confirmed metabolites of condensation or coupling reactions of all of these components with phenol and/or catechol and possibly other fragments identified using GS-MS.

**Figure 7:** The GC-MS fragmentation profile of the major peaks identified; a) control (phenol); b) standard (catechol).

**Figure 8:** The hypothesized phenol biodegradation mechanism, which revealed: the sample's catechol-2,3-dioxygenase pathway.

Several researchers have identified single bacterial strains with high phenol removal efficacy, such as *C. flaccumfaciens* [66, 70, 71, 72]. *C. flaccumfaciens*, on the other hand, possesses two of the four plant growth-promoting traits in addition to being a phenol biodegrader. *C. flaccumfaciens* had a high yield factor and tolerance to phenol when compared to other strains of bacteria. The maximum specific growth rate (μmax) of *C. flaccumfaciens* occurred at an initial phenol concentration of 291 mg/L, which is higher than those of *Rhodococcus* sp. Strain SKC [50, 73], *Bacillus cereus* MTCC 9817 [71], Mixed culture [74], *Pseudomonas* WUST-C1 [75] and *Alcaligenes faecalis* [76] for almost the same phenol concentration range. These findings show that *C. flaccumfaciens* has a higher tolerance and adaptation to phenol than any other bacteria, indicating its potential for rhizoremediation and crop yield preservation in phenol-stressed conditions.

## 4 Conclusion

*C. flaccumfaciens*, a characterized plant growth stimulating bacterium, was utilized to assess the growth kinetics and biodegradation of phenol. Haldane's growth kinetics inhibition coefficient (Ki), half-saturation coefficient (Ks), and the maximum specific growth rate (max) for phenol-dependent growth kinetics were calculated using the Haldane inhibition model and were estimated to be 329 (mg/L), 9.14 (mg/L), and 1.05 (h^−1^), respectively. The Haldane equation is well suited to empirical data, with a sum of squared error (SSR) of 1.36 × 10^−3^. The modified Gombertz model also forecasts phenol biodegradation trends with high accuracy. *C. flaccumfaciens'* potential to biodegrade phenol and enhance synchronous plant growth was identified in this investigation. In phenol-stressed circumstances, this could help with rhizoremediation and crop yield preservation.

## Declarations

### Author contribution statement

Khaled Khleifat; Mousa Magharbeh; Moath Alqaraleh & Mutaz Al-Sarayrah: Conceived and designed the experiments; Performed the experiments; Analyzed and interpreted the data;

Contributed reagents, materials, analysis tools or data; Wrote the paper.

Ibrahim Alfarrayeh; Yaseen Al Qaisi; Ahmad Alsarayreh & Mohammad Alkafaween: Performed the experiments; Analyzed and interpreted the data; Wrote the paper.

### Funding statement

Khaled M. Khleifat was supported by Deanship of Scientific Research at Mutah university/Jordan [316/2020].

### Data availability statement

Data will be made available on request.

### Declaration of interests statement

The authors declare no conflict of interest.

### Additional information

No additional information is available for this paper.
